# Involvement of Ca^2+^-activated K^+^ channel 3.1 in hypoxia-induced pulmonary arterial hypertension and therapeutic effects of TRAM-34 in rats

**DOI:** 10.1042/BSR20170763

**Published:** 2017-07-27

**Authors:** Shujin Guo, Yongchun Shen, Guangming He, Tao Wang, Dan Xu, Fuqiang Wen

**Affiliations:** 1 Laboratory of Pulmonary Diseases and Department of Respiratory Medicine, West China Hospital of Sichuan University, Chengdu, Sichuan 610041, China; 2 The Affiliated Hospital of University of Electronic Science and Technology of China, Internal Medicine of Sichuan Academy of Medical Sciences and Sichuan Provincial People’s Hospital, Chengdu, Sichuan 610072, China

**Keywords:** ERK, p38, hypoxia, Kca3.1, pulmonary arterial hypertension, pulmonary vascular remodeling, TRAM-34

## Abstract

Pulmonary artery hypertension (PAH) is an incurable disease associated with the proliferation of pulmonary artery smooth muscle cells (PASMCs) and vascular remodeling. The present study examined whether TRAM-34, a highly selective blocker of calcium-activated potassium channel 3.1 (Kca3.1), can help prevent such hypertension by reducing proliferation in PASMCs. Rats were exposed to hypoxia (10% O_2_) for 3 weeks and treated daily with TRAM-34 intraperitoneally from the first day of hypoxia. Animals were killed and examined for vascular hypertrophy, Kca3.1 expression, and downstream signaling pathways. In addition, primary cultures of rat PASMCs were exposed to hypoxia (3% O_2_) or normoxia (21% O_2_) for 24 h in the presence of TRAM-34 or siRNA against Kca3.1. Activation of cell signaling pathways was examined using Western blot analysis. In animal experiments, hypoxia triggered significant medial hypertrophy of pulmonary arterioles and right ventricular hypertrophy, and it significantly increased pulmonary artery pressure, *Kca3.1* mRNA levels and ERK/p38 MAP kinase signaling. These effects were attenuated in the presence of TRAM-34. In cell culture experiments, blocking Kca3.1 using TRAM-34 or siRNA inhibited hypoxia-induced ERK/p38 signaling. Kca3.1 may play a role in the development of PAH by activating ERK/p38 MAP kinase signaling, which may then contribute to hypoxia-induced pulmonary vascular remodeling. TRAM-34 may protect against hypoxia-induced PAH.

## Introduction

Pulmonary artery hypertension (PAH), defined as elevated pulmonary artery pressure, occurs in several diseases, such as idiopathic PAH, end-stage chronic obstructive pulmonary disease (COPD), asthma, and lung fibrosis. PAH is diagnosed using hemodynamic measurements obtained via right heart catheterization or echocardiography; the condition is defined as mean pulmonary artery pressure ≥25 mmHg at rest or ≥30 mmHg during movement [1].

Despite its diverse causes, PAH appears to be driven usually by vasoconstriction [2,3] and vascular remodeling. Various stimuli, including hypoxia, may contribute to PAH initiation: small-animal studies have associated PAH with proliferation of pulmonary artery smooth muscle cells (PASMCs) in small intrapulmonary arteries; leading to inflammatory cell infiltration into the lung, ultimately inducing the release of numerous mediators of pulmonary vessel remodeling [4]. Although PAH has been associated with pathways mediated by endothelin, nitric oxide, and prostacyclin [5], targetted pathways’ drugs often fail to alleviate the gradual increase in pulmonary pressure [6]. Lung transplantation is an option for only a fraction of patients [7]. Thus, despite therapeutic advances against PAH in small animals [8,9] and humans [10], standard treatments cannot cure the disease and improve quality of life or prognosis. Researchers continue to search for antihypertensive and antiproliferative treatments that can prevent or reverse medial thickening as well as PASMC hypertrophy and hyperplasia [11].

One possibility is to block K^+^ channels, since cell proliferation requires increased expression of such channels [12–14]. Calcium (Ca^2+^)-activated K^+^ channel 3.1 (Kca3.1) is widely expressed in non-neuronal tissues, including epithelia, endothelia, and smooth muscle, where it regulates intracellular Ca^2+^ concentration and membrane potential [15]. Blocking Kca3.1 with the highly selective blocker TRAM-34 [16] can reduce cell proliferation in cancer [17], angiogenesis, post-interventional arterial restenosis, atherosclerosis, and asthma [18]. Our group has shown that treating PASMC cultures with TRAM-34 can inhibit hypoxia-induced proliferation [19]. In the present study, we wanted to examine whether this *in vitro* effect would translate into therapeutic effects against hypoxia-induced PAH *in vivo*.

In addition, we wanted to begin to understand the molecular pathways by which hypoxia and TRAM-34 exert opposite effects on the pulmonary artery, as well as clarify how Kca3.1 fits into this picture. We focussed on mitogen-activated protein kinases (MAPKs) because they regulate cell proliferation and differentiation after exposure to hypoxia. Hypoxia reduces intracellular Ca^2+^ concentrations, which may activate MAPKs and lead to cellular proliferation and differentiation [20]. In particular, p38 and ERK1/ERK2 kinases participate in vascular and non-vascular smooth muscle cell contraction [21], and p38 MAPK regulates ET-1-induced contraction of pulmonary artery in dogs [22,23]. Inhibiting p38 MAPKs reverses hypoxia-induced dysfunction in pulmonary artery endothelium [24].

Given this literature, we hypothesized that hypoxia activates the Kca3.1 channel and downstream ERK/p38 MAPK signaling, leading to PAH. We also hypothesized that TRAM-34 would partially reverse these effects, thereby ameliorating hypoxia-induced PAH.

## Methods

### Animals and treatments

Animal experiments were approved by the Animal Ethics Committee of Sichuan University, and procedures conformed to the National Institutes of Health Guide for the Care and Use of Laboratory Animals.

Thirty-six male Sprague–Dawley rats (350–400 g) were equally divided into six groups (A: normoxia, B: normoxia in the presence of 300 μg/kg TRAM-34, C: normoxia in the presence of 600 μg/kg TRAM-34, D: hypoxia, E: hypoxia in the presence of 300 μg/kg TRAM-34, F: hypoxia in the presence of 600 μg/kg TRAM-34) and then exposed to room air (21% O_2_) or chronic hypoxia (10% O_2_) for 3 weeks using a ProOx P110 oxygen controller (BioSpherix, NY, U.S.A.). The concentration of O_2_ was maintained at 10% by regulating the flow of compressed nitrogen (N_2_). Starting on the first day of hypoxia, a subset of animals in each type of atmosphere received intraperitoneal injections of TRAM-34 daily (1-[(2-chlorophenyl)diphenylmethyl]-1H-pyrazole, Sigma–Aldrich, St. Louis, MO) at doses of either 300 or 600 μg/kg.

### Measurement of pulmonary artery pressure and cardiac chamber size

Animals were anesthetized using pentobarbital sodium, the right internal jugular vein was surgically separated, and a home-made polyethylene pressure transducer was cannulated into the pulmonary artery through the right ventricle. Pulmonary artery pressure was measured and once pressure waveforms had stabilized, the pressure was measured continuously using a BL420 Data Acquisition and Analysis System (Chengdu TME Technology, Chengdu, China).

At the end of the experiment, rats were killed with pentobarbital sodium anesthesia, and the hearts were collected. The right ventricle, left ventricle, and septum were carefully separated and weighed. A right ventricular hypertrophy index (RVHI) was calculated from the formula [25]: RVHI = right ventricle weight/(left ventricle weight + septum weight).

### Lung histology

The right lung was processed for histology and the left lung for biochemistry (see section on ‘Western blot analysis’ below). We ligated the left main-stem bronchus, instilled the right lung with 4% polyformaldehyde (pH 7.4) for 30 min, and then clipped the right lung. All right lungs were fixed in 4% polyformaldehyde, paraffin-embedded, sliced into sections 4-μm thick, and stained with Hematoxylin and Eosin. The left lung was cut and preserved in liquid nitrogen for biochemical analysis.

To evaluate the morphology of muscularized pulmonary artery, the medial wall thickness (MWT) with vessel diameter of 100 μm was assessed by the formula: MWT = (medial thickness × 2/external diameter) × 100% [26].

### Culturing PASMCs

Primary PASMCs were isolated as described [27]. Briefly, intrapulmonary arteries were separated and excised, and endothelial cells were removed by scraping. The pulmonary arteries were cut into pieces and incubated in Dulbecco’s minimum Eagle's medium (DMEM) containing 10% FBS, 100 U/ml penicillin, and 0.1 mg/ml streptomycin. Tissue explants were discarded after 7 days, and the remaining PASMCs were incubated in culture medium containing 20% FBS until they reached 90% confluence. Cells were digested with 0.05% trypsin in PBS, then subcultured in medium containing 10% FBS. PASMCs were identified based on immunostaining with a polyclonal antibody against rat α-smooth muscle actin.

### Exposure of PASMCs to hypoxia

PASMC cultures from passages 5–7 were starved in DMEM containing 0.2% FBS for 24 h, then subjected for 24 h either to normoxia (21% O_2_ and 5% CO_2_) or hypoxia (3% O_2_ and 5%CO_2_). Oxygen concentration in the chamber was verified using an oxygen sensor (BioSpherix). Our hypoxia conditions were similar to those of other studies, which typically exposed the cells to 0–10% O_2_ for 4–24 h.

### Treatment of PASMCs with TRAM-34 or Kca3.1 siRNA

When PASMCs reached 90% confluence, cells were cultured in six-well dishes. PASMCs were treated with TRAM-34 at doses of 100 or 200 nM for 24 or 48 h. For siRNA transfection, cells were transfected with purified fragment siRNA targetting Kca3.1 (5′-GCCAAACUAUACAUGAACA-3′, synthesized by Ribobio, China) at different concentrations (25, 50, or 100 μM) and action times (24, 48, or 72 h). Transfection was carried out using INTERFERin (Polyplus, France) according to the manufacturer’s instructions.

### Assay of Kca3.1 expression

RNA was extracted from PASMC cultures and left lungs of rats that had been treated or transfected as described above. Extraction was performed using TRIzol (Invitrogen, Carlsbad, CA, U.S.A.), and cDNA was synthesized by MMLV reverse transcriptase (MBI Fermentas, Ontario, Canada). This cDNA was quantitated by PCR in a Bio–Rad iCycler CFX using SYBR1 GreenER qPCR SuperMix (Bio–Rad, U.S.A.) and primers targetting regions in the genes encoding Kca3.1 and β-actin. Primers and PCR conditions were as described in [19].

### Western blot analysis of MAPK levels

Total protein was extracted from right lung tissue from rats and PASMC cultures treated or transfected as described above, and resulting protein concentrations were assayed using the BCA method. Equal amounts of protein (20 μg) were electrophoresed on an SDS/polyacrylamide gel (12% gel), and then electroblotted on to PVDF membrane. Membranes were blotted with primary antibodies (CST, U.S.A.) against t-p38 MAPK (1:2000), p-p38 MAPK (1:1000), t-ERK MAPK (1:2000), or p-ERK MAPK (1:1000). As a loading control, membranes were blotted with antibody against tubulin (1:2000; Epitomics, U.S.A.). Then membranes were blotted with a horseradish peroxidase–conjugated secondary antibody (1:4000; Epitomics, U.S.A.) and stained using the Clarity ECL Western Blot Substrate (Bio–Rad, U.S.A.).

### Statistical analysis

Values are expressed as mean ± S.D., and data were analyzed statistically using SPSS 13.0 (Chicago, U.S.A.). Differences between treatment groups were assessed for significance using one-way ANOVA and Tukey’s HSD test. The threshold for significance was defined as *P*<0.05.

### Ethics

The animal experiments in the present study were approved by the Animal Ethics Committee of Sichuan University. Procedures conformed to the National Institutes of Health Guide for the Care and Use of Laboratory Animals, as well as to all relevant institutional and national guidelines and regulations.

## Results

### TRAM-34 administration attenuated hypoxia-induced pulmonary artery remodeling, pulmonary artery pressure, and RVHI in rats

Exposure to hypoxia for 3 weeks led to thick-walled pulmonary arteries with media hyperplasia, which was not observed in control animals (Figure 1). Hypoxia also significantly increased RVHI (Figure 2A); it increased pulmonary artery pressure, consistent with severe PAH (Figure 2B); and it increased medial wall thickness of arterioles, indicating pulmonary artery remodeling (Figure 2C). However, TRAM-34 intervention could ameliorate hypoxia-induced PAH, decrease RVHI, and inhibit MWT in rats, and these results showed that Kca3.1 played important role in PAH pathogenesis.

**Figure 1:** Lung sections from rats exposed for 3 weeks To (**A**) normoxia, (**B**) normoxia in the presence of 300 μg/kg TRAM-34, (**C**) normoxia in the presence of 600 μg/kg TRAM-34, (**D**) hypoxia, (**E**) hypoxia in the presence of 300 μg/kg TRAM-34, or (**F**) hypoxia in the presence of 600 μg/kg TRAM-34. Sections were stained with Hematoxylin and Eosin. In all the images, vessel diameter was 100 μm. Magnification: 20×.

**Figure 2:** Hypoxia-induced changes In (**A**) RVHI, (**B**) pulmonary artery pressure, and (**C**) MWT. Rats were exposed to normoxia or hypoxia in the absence or presence of 300 μg/kg TRAM-34 or 600 μg/kg TRAM-34. ^#^*P*<0.05 compared with normoxia group; ^##^*P*<0.05 compared with hypoxia group.

### Up-regulation of Kca3.1 expression in hypoxia-exposed lungs and PASMCs

To evaluate that Kca3.1 is involved in hypoxia-induced pulmonary artery remodeling and PAH, levels of *Kca3.1* mRNA were compared between lungs from hypoxia-exposed rats and control animals. *Kca3.1* mRNA levels were higher in hypoxia-exposed animals (Figure 3A).

**Figure 3:** *Kca3.1* mRNA levels after TRAM-34 and Kca3.1 siRNA intervention (**A**) *Kca3.1* mRNA expressions were measured in rats treated as described in Figure 2. (**B**) *Kca3.1* mRNA levels after TRAM-34 intervention at dose of 100 or 200 nM in PASMCs. (**C**) *Kca3.1* mRNA expressions after 50 μM Kca3.1 siRNA transfection. ^#^*P*<0.05 compared with normoxia group; ^##^*P*<0.05 compared with hypoxia group.

Our recent results showed that TRAM-34 could ameliorate PASMCs proliferation at doses of 100 and 200 nM after 24 h of hypoxia exposure [19], then we used these dosages and action times for *in vitro* experiments. The results showed that *Kca3.1* mRNA levels decreased after TRAM-34 intervention (Figure 3B).

For the siRNA transfection, the pre-experiments found that PASMCs transfected with 50 μM Kca3.1 siRNA for 24 h could significantly inhibit cell proliferation. *Kca3.1* mRNA levels were decreased after siRNA transfection (Figure 3C).

### TRAM-34 administration reduced hypoxia-induced ERK MAPK signaling in rat lungs

To determine whether MAPKs are involved in hypoxia-induced PAH, we compared levels of ERK/p38 MAPK signaling in lungs of hypoxia-exposed rats and control animals. Hypoxia was associated with higher levels of p-ERK and p-p38, while levels of t-ERK and t-p38 remained unchanged (Figure 4). These increases in p-ERK and p-p38 were much smaller in the presence of TRAM-34, which did not affect levels of t-ERK and t-p38. These results suggest that Kca3.1 regulates hypoxia-induced pulmonary artery proliferation via the p-ERK/p38 signaling pathway.

**Figure 4:** Signaling proteins expression in rat lungs after TRAM-34 intervention (dosage: 300 or 600 μg/kg) ^#^*P*<0.05 compared with normoxia group; ^##^*P*<0.05 compared with hypoxia group.

### Inhibition of Kca3.1 using TRAM-34 or siRNA-reduced, hypoxia-induced ERK/p38 MAPK signaling in PASMC cultures

Since proliferation of PASMCs is a dominant contributor to PAH, rat primary PASMCs were isolated and cultured for proliferative experiment. To further validate the role of Kca3.1 in hypoxia-induced pathology, TRAM-34 and Kca3.1 siRNA were administered separately to PASMCs for 24 h simultaneously. Kca3.1 siRNA transfection for 24 h could suppress *Kca3.1* mRNA in PASMCs under both hypoxia and normoxia conditions (Figure 3C). Both pharmacological and siRNA interventions decreased p-ERK and p-p38 expression, with no effect on t-ERK and p-p38, consistent with the results observed *in vivo* (Figure 5).

**Figure 5:** Signaling proteins expression in PASMCs after TRAM-34 intervention (dosage: 100 or 200 nM) and 50 μM Kca3.1 siRNA transfection ^#^*P*<0.05 compared with normoxia group; ^##^*P*<0.05 compared with hypoxia group.

## Discussion

The results of the study mainly demonstrated that hypoxia exposure significantly increased the wall thickness of rat pulmonary arterial, PAP, and RVHI as well as *Kca3.1* mRNA and protein levels. TRAM-34 intervention markedly reduced the pulmonary artery remodeling, PAP, and RVHI that were caused by hypoxia exposure. Furthermore, TRAM-34 decreased p-ERK and p-p38 expression induced by hypoxia.

We have already demonstrated that TRAM-34 decreases hypoxia-induced rat PASMC proliferation and hypoxia-stimulated Kca3.1 expression *in vitro* [19]. Consistent with our *in vitro* study results, Kca3.1 expression were significantly higher in the hypoxia group than in the normoxia group. Both TRAM-34 and Kca3.1 siRNA could decrease hypoxia-induced p-ERK and p-p38 overexpression. Our results suggest a possible role of TRAM-34 in the attenuation of hypoxia-induced pulmonary artery remodeling and PAH.

It has been reported that in rats exposed to chronic hypoxia for 3 weeks, there was an increase in right ventricular systolic pressure (RVSP) and enhanced muscularization of small pulmonary arteries [28]. Similarly, elevated RVSP and increased pulmonary vessels muscularization have also been detected in rats after 3 or 5 weeks of hypoxia exposure. Both RVSP and PAP were major indexes for evaluation of elevated PAH [7–9]. Consistent with these findings, in our study, 3 weeks of hypoxia exposure induced remarkable thickness of the pulmonary artery medial wall and significantly increased PAP in rats. These results suggest that hypoxia may act as a leading role in pulmonary artery remodeling and PAH.

Potassium channels are widely distributed in artery walls, and are essential for membrane potential maintenance, cell volume, migration, proliferation, and apoptosis [12]. Calcium-activated potassium channels is a group of potassium channels, including large conductance Ca^2+^-activated K^+^ channels (Bkca), intermediate conductance Ca^2+^-activated K^+^ channels (Kca3.1), and small conductance Ca^2+^-activated K^+^ channels (Skca) [15]. Calcium activated potassium channels contribute to the pathogenesis of PAH, especially the Kca3.1 [29]. It has been found that Bkca on smooth muscle cells are transformed to Kca3.1 to promote cell migration and proliferation [29]. Kca3.1 acts as a regulator in the proliferative switch. For example, human endometrial cancer could be inhibited by blocking the Kca3.1 [16]; balloon catheter delivery of TRAM-34 locally could prevent coronary artery VSMC phenotypic switching and reduce subsequent restenosis [30]; benign prostatic hyperplasia could be suppressed by blockage of Kca3.1 [31], and renal fibrosis is significantly attenuated by targetted interference of Kca3.1. TRAM-34 is a derivative of triarylmethane clotrimazole, and exerts highly selective block role to Kca3.1 [13]. Since Kca3.1 plays a key role in converting proliferation, we hypothesized that hypoxia exposure may increase Kca3.1 expression, and blocking the Kca3.1 channel could suppress hypoxia-induced PAH. In the present study, we found a marked elevation in Kca3.1 expression both *in vivo* and *in vitro* compared with those from the control group. Administration of TRAM-34 intra peritoneal injections decreased hypoxia-induced PAP, RVHI, and vascular remodeling.

Kca3.1 is an important regulator of the Ca^2+^-dependent proliferation mechanisms in VSMC [32]. Recently, it is becoming increasingly clear that control of ion channels in the transcriptional process contributes to the phenotypic modulation of both the differentiated and the proliferative phenotype in VSMC [33,34]. Up-regulation of the intermediate-conductance Ca^2+^-activated K^+^ channel, Kca3.1, and store-operated Ca^2+^ channels have been linked with the proliferative phenotype [35,36]. Blockage of Kca3.1 with TRAM-34 prevents down-regulation of myocardin and smooth muscle myosin heavy chain, thus promoting the differentiated phenotype and suppressing the proliferative one [36,37]. In recent work [19], we showed that both TRAM-34 and siRNA against Kca3.1 decrease hypoxia-induced PASMC proliferation *in vitro*, consistent with the *in vivo* experiments.

Since Kca3.1 helps to determine intracellular Ca^2+^ concentrations and this is important for Ras/ERK and Ras/Raf/MEK/ERK signaling pathways [14,38], we examined whether the ERK/p38 MAPK pathway may mediate the observed ability of TRAM-34 to alleviate PAH in rats. We found that hypoxia elevated levels of p-ERK and p-p38, while TRAM-34 reduced them. Our results suggest that ERK/p38 MAPK signaling plays an important role in PAH and is a promising therapeutic target. Our findings are consistent with the known role of these kinases in regulating cell proliferation and differentiation in response to stimuli such as hypoxia, and in regulating contraction of vascular and non-vascular smooth muscle cells [21]. In fact, one study suggests that p38 MAPK mediates the sustained pulmonary artery contraction induced by hypoxia in rats [24].

The effect of acute hypoxia on vascular remodeling is investigated by the culture of PASMCs. Hypoxia is generally conducted for 4–24 h in 0–10% O_2_ with measurement of cell proliferation [38]. Hypoxia (1–5% O_2_) was positively correlated with acute hypoxia and PASMC proliferation [39]. Accordingly, we chose 3% O_2_ for 24 h for PASMC hypoxia. Both TRAM-34 and siRNA administration could decrease hypoxia-induced proliferation, and these results are concomitant with those of an animal experiment.

In summary, hypoxia exposure significantly induced pulmonary artery remodeling, PAP elevation, and increased expression of Kca3.1. TRAM-34 administration effectively attenuated the hypoxia-induced pulmonary arterial remodeling and PAH, and reduced p-ERK and p-p38 expression. Kca3.1 transfected with siRNA *in vitro* decreased rat PASMC proliferation induced by hypoxia exposure. These results suggest that TRAM-34 could attenuate hypoxia-induced PAH through the ERK/p38 MAPK pathway.

## Abbreviations

Bkca: large conductance Ca^2+^-activated K^+^ channel
CST: cell signaling technology
ERK: extracellular regulated protein kinase
ET-1: endothelin-1
HSD: honestly significant difference
Kca3.1: calcium-activated potassium channel 3.1
MAPK: mitogen-activated protein kinase
MMLV: Moloney murine leukemia virus
MWT: medial wall thickness
PAH: pulmonary artery hypertension
PAP: pulmonary artery pressure
PASMC: pulmonary artery smooth muscle cell
RVHI: right ventricular hypertrophy index
RVSP: right ventricular systolic pressure
SKca: small conductance Ca^2+^-activated K^+^ channel
t-P38: total-P38
t-ERK: total-extracellular regulated protein kinase
VSMC: vascular smooth muscle cell
